The article "Revealing PAK2's Function in the Cell Division through MKLP1's Interactome" was retracted in 2024. Reasons: signs of a paper mill; suspected computer-generated content; unreliable results or conclusions; concerns about the data.

# Revealing PAK2's Function in the Cell Division through MKLP1's Interactome

**DOI:** 10.1155/2020/8854245

**Published:** 2020-11-06

**Authors:** Zhao-huan Zhang, Xiu-ling Liu, Yun-yi Zhu, Hai Huang, Xiao-hui Xu

**Affiliations:** ^1^School of Life Sciences, Shanghai University, Shanghai 200444, China; ^2^Department of Neurology, Changzheng Hospital, Naval Medical University, Shanghai 200433, China; ^3^School of Preclinical Medicine, Wannan Medical College, Wuhu 241001, China

## Abstract

Cell division-related proteins are essential for the normal development and differentiation of cells and may be related to the occurrence of cancer and the drug resistance mechanism of cancer cells. The mitotic kinesin-like protein 1 (MKLP1) is a kinesin protein that has been involved in the assembly of the midzone/midbody during mitosis and cytokinesis. In this study, we found that the tail domain of MKLP1 exhibited an autoinhibitory effect on its motor activity. Overexpression of the tail domain in HEK293 cells blocked cytokinesis and caused bi-/multinucleation. It is possible that protein binding to the MKLP1 tail relieves this autoinhibition and induces the motility of MKLP1. We used the GST pull-down assay followed by the LC-MS/MS analysis and identified 54 MKLP1 tail domain-specific binding proteins. Further, we confirmed the MS result by coimmunoprecipitation and FRET that a serine/threonine kinase, p21-activated kinase 2 (PAK2), binding to MKLP1. Endogenous PAK2 expression was found to be identical to that of MKLP1 in HEK293 cells during cytokinesis. Finally, functional studies indicated that when PAK2 expression was downregulated by siRNA, MKLP1 underwent a change in its localization away from the midbody, and cell cytokinesis was subsequently impeded. This study presents a novel regulatory mechanism that PAK2 promotes the activation of MKLP1 and contributes to complete cell cytokinesis.

## 1. Introduction

Proper cell division requires spatiotemporal coordination of cytoplasmic division (cytokinesis) and nuclear division (mitosis) to ensure that each daughter cell receives a complete chromosome and proper cytoplasmic and organelle components. Cell division-related protein dysregulations are related to the occurrence of cancer and the drug resistance mechanism of cancer cells. MKLP1 is an important kinesin involved in cell division, and its regulatory mechanism is not yet clear. The depletion of MKLP1 function by microinjection of MKLP1 antibodies in mammalian cells inhibits midbody formation and completion of cytokinesis. Moreover, overexpression of an ATP-binding mutant of MKLP1 inhibits the completion of cytokinesis and caused bi-/multinucleation [1]. These results indicate that the motor activity of MKLP1 is necessary for the completion of cytokinesis.

We have previously reported that the tail domain of MKLP1 is necessary for the dendritic localization of MKLP1 [2]. Here, we found that tail domain-deleted MKLP1 mutants have increased motility. Furthermore, we found that overexpression of the tail domain of MKLP1 in HEK293 cells inhibits the completion of cytokinesis and causes bi-/multinucleation. This finding suggests that the tail domain of MKLP1 exhibited autoinhibition on its motor activity like the other kinesin proteins [3–6]. It could be predicted that any protein binding to the tail domain would relieve the inhibition of MKLP1's tail domain on its ATP-binding activity and would contribute to the motility of MKLP1, finally facilitating cytokinesis. To identify regulatory partners of MKLP1, we used GST pull-down and MALDI-TOF mass spectrometry analysis to screen for proteins associated with the MKLP1 tail domain. The results demonstrated that PAK2, a member of the family of serine/threonine kinases, bound to the MKLP1 tail. Immunocytochemistry examination proved that MKLP1 and PAK2 shared an identity in the temporal and spatial expressions at the midbody during cytokinesis, and a direct interaction was further confirmed by FRET and coimmunoprecipitation assay. Finally, by RNA-interference-mediated knockdown of PAK2 expression, we proved that PAK2 was involved in cell cytokinesis, perhaps through its regulatory effect on MKLP1 localization.

## 2. Materials and Methods

### 2.1. Cell Culture and Synchronization

HEK 293 cells were cultured in DMEM supplemented with 10% fetal bovine serum (FBS) (Gibco™, Invitrogen, Carlsbad, CA, USA). To obtain cells synchronized at cytokinesis, HEK 293 cells were grown on coverslips and treated with 2.5mM thymidine (Sigma) for 12-16 hours. The cells were then washed with PBS and incubated for 5 hours in a fresh culture medium. Next, nocodazole (Sigma) was added to the medium to a final concentration of 0.05*μ*g/ml. For another 6 hours, cells were washed with 0.01M PBS and incubated for an additional 8 hours in a fresh culture medium. Finally, the cells were fixed at various time points thereafter for immunofluorescence analysis.

#### 2.1.1. Plasmid Construction

The sequences of small interfering RNA targeting *PAK2* were as follows: siPAK2: 5′-GAAACTGGCCAAACCGTTAT-3′ [7] and nonsilent sequence (scramble): 5′-GAAAGTCCCGATACCGATAT-3′. For the generation of shRNA expression vectors, small hairpin RNAs (shRNAs) against PAK2 and scrambled shRNA were designed according to the above sequences and were chemically synthesized by GenePharma Co., Ltd. (Shanghai, China) with the following sequences: shPAK2: 5′-GATCCGAAACTGGCCAAACCGTTATTCAAGAGATAACGGTTTGGCCAGTTTCTTTTTTA-3′ and scramble: 5′-GATCCGAAAGTCCCGATACCGATATTCAAGAGATATCGGTATCGGGACTTTCTTTTTTA-3′. The sequences form a loop by hydrogen bonding of AT or GC. The oligonucleotides were subcloned into the *Bam*HI and *Hin*dIII sites of the pGPU6/GFP/Neo vector. Human PAK2 cDNA was generated by RT-PCR amplification from HEK293 cell cDNA. PAK2 cDNA was then cloned into the pEYFP-N1 vector. To rescue PAK2 knockdown, we also synthesized an RNAi-resistant isoform of human PAK2. Five nucleotides in the siRNA targeting sequence were changed and subcloned into PCDNA3.1 plasmid. The MKLP1 mutants were generated as previously reported [2]. pGEX-4T1-MKLP1-TD (GST-MKLP1-TD) is generated by a subclone MKLP1 tail domain (AA600-856) inserted to the pGEX-4T1 vector. All constructs were confirmed by DNA sequencing.

#### 2.1.2. GST Protein Expression and Purification

GST protein expression and purification methods are the same as we previously reported [8]. GST-MKLP1-TD fusion or GST proteins were expressed in Ecoli BL21 (DE3) cells. The bacterial culture was induced with 0.2mM IPTG at 25°C for 6h and then centrifuged in 2 × 250mL volumes at 3500g for 10min at 4°C. The bacterial pellets were resuspended in 12mL each of lysis buffer with 1mM PMSF, 5mM DTT, and 0.5% *v*/*v* Triton X-100. Samples were then incubated on ice for 30 min and centrifuged at 12000g for 30min at 4°C. Then, the supernatants were incubated with 1mL of a 50% *v*/*v* glutathione-Sepharose bead for 1 hour at 4°C. Next, the samples were centrifuged at 5000g for 1min at 4°C, and the supernatants were discarded. The pellets were washed by 20mL of PBS (pH7.4) followed by centrifugation at 5000g for 1min at 4°C. The pellets were washed 3 times in 1mL of wash buffer with a protease inhibitor at room temperature. Protein concentration was determined by a Lowry assay.

#### 2.1.3. GST Pull-Down Assay/Mass Spectrometry and the Data Analysis

The GST pull-down assay and mass spectrometry and the data analyses are the same as previously reported [8, 9].

#### 2.1.4. Gene Transfection

HEK293 cells were grown on glass coverslips until they reached 70-80% confluence. Purified plasmids were then transfected into the HEK293 cells using Lipofectamine 2000 (Invitrogen) following the manufacturers' instructions. After 48 hours, cells were washed with 0.01M PBS and fixed.

#### 2.1.5. Immunofluorescence Microscopy

HEK293 cells were fixed for 30-45min with 4% paraformaldehyde at room temperature. Fixed cells were permeabilized with 0.1% Triton X-100 (30min) and blocked with 1% bovine serum albumin and then incubated at 4°C overnight with primary antibody (rabbit polyclonal anti-PAK2(#2608), 1 : 100, Cell Signaling Technology; rabbit polyclonal anti-MKLP1 (N-19), 1 : 100, Santa Cruz, CA), and then, proteins were detected using Cy3-conjugated second antibodies (1 : 500, Jackson ImmunoResearch). To visualize DNA, cells were incubated for 2-5min with 1 *μ*g/mL DAPI. Microscopic images were captured using Nikon Eclipse TE2000 inverted microscope equipped with epifluorescence optics.

#### 2.1.6. Immunoprecipitation and Immunoblotting

Cultured HEK293 cells were lysed in RIPA buffer supplemented with 0.5 mM PMSF and Protease Inhibitor Cocktail (Roche), and then, the lysed cells were incubated on ice for another 20 minutes. Next, lysates were subjected to centrifugation at 12000g for 20-30minutes at 4°C. The supernatant (almost 500*μ*L) was incubated with 5*μ*L of the first antibody for 2 hours at 4°C. Protein G-agarose beads (Roche) were added for 12 hours at 4°C. The immunoprecipitated beads were washed three times in a lysis buffer then boiled for 5 minutes in a loading buffer. Western blotting was then performed.

#### 2.1.7. Fluorescence Resonance Energy Transfer (FRET) Measurements with Three-Channel Microscopy

Following the method we used previously [9, 10], HEK293 cells were plated on glass coverslips and were transfected with pEYFP-PAK2 and pECFP-MKLP1. The cells were then cultured for another 24 hours. The images were taken using an Olympus IX71 inverted microscope with a 60x oil objective lens (NA = 1.45) and cooled CCD Cascade 512F (roper). For imaging, Image-Pro Plus® version 5.0.1 software (Media Cybernetics) was used. The filter sets used were YFP (excitation, 500/25nm; emission, 545/35nm), CFP (excitation, 440/21nm; emission, 480/30nm), and FRET (excitation, 440/21nm; emission, 535/26nm). The FRET ratio was calculated on a pixel-by-pixel basis for the entire image using the following equation: FRETratio(FR) = [FRET − (*b* × CFP)]/(*a* × YFP), where FRET, YFP, and CFP correspond to background-subtracted images of cells coexpressing CFP and YFP acquired through the FRET, YFP, and CFP channels, respectively. The parameters “a” and “b” are the fractions of the bleedthrough of YFP and CFP fluorescence through the FRET filter channel, respectively. In our system, *a* = 0.090 ± 0.0065 and *b* = 0.75 ± 0.013.

## 3. Results and Discussion

### 3.1. The Tail Domain of MKLP1 Affects the Motility of MKLP1

MKLP1 is a kinesin-like motor protein. MKLP1 can move along microtubules to the spindle midzone and the cleavage furrow during anaphase, finally concentrating at the midbody during cytokinesis and executing its normal function during cell division [11]. Thus, the motility of MKLP1 is needed for its function in cytokinesis. Microtubules are usually anchored their minus end in the centrosome and their plus end extending toward the cell periphery. MKLP1 is a plus end-directed microtubule motor, and active MKLP1 tends to move along microtubules toward the periphery of the cell which the microtubule plus end is located. The motility of MKLP1 can be predicted by detecting its localization in cells. We generated the two tail domain-deleted mutants (*Δ*C16-MKLP1-GFP and MSD-MKLP1-GFP) as shown in Figure 1(a), and the subcellular localization was assessed by overexpression in HEK293 cells. As shown in Figure 1(b), full-length MKLP1 did not associate with microtubules and was concentrated to the nucleus, indicating that full-length MKLP1 motor activity is inhibited. Both tail domain-deleted mutants (*Δ*C16-MKLP1-GFP and MSD-MKLP1-GFP) tended to associate with microtubules and accumulate at the periphery of the cell, indicating their increased motor activity. As kinesin motors use the energy derived from ATP hydrolysis to move along microtubules, the motility of MKLP1 is also ATP dependent [11]. Additional experiments were performed to test the effect of the tail domain on the ATP binding site. As shown in Figure 1(a), the ATP binding point GKT-AAA (117–119) was mutated in addition to the tail domain deletion, resulting in the mutants ΔC16'-MKLP1-GFP and MSD'-MKLP1-GFP, which can bind with microtubules but cannot maintain their localization at the periphery of the cell (Figures 1(b) and 1(c)). These results indicated opposing roles for the tail domain and ATP-binding domain in MKLP1 motility. To determine whether overexpression of the tail domain of MKLP1 inhibits the completion of cytokinesis, we generated eGFP fusion constructs of the tail domain (TD-MKLP1) and eGFP fusion constructs of the stalk and tail domain (STD-MKLP1) as shown in Figure 1(a). HEK293 cells were transfected with these two constructs, and a vacant vector was used in parallel as a control. Two days later, the cellular phenotype was analyzed. Cells overexpressing either TD-MKLP1 or STD-MKLP1 showed an increase in the number of bi-/multinucleated cells compared with the control (Figures 1(d) and 1(e)). In accordance with the idea that MKLP1's motility is necessary for correct cell division, our results suggested that overexpression of the MKLP1 tail domain, which seems to act as a dominant-negative competitor for endogenous MKLP1, impeded the endogenous MKLP1 function of facilitating cytokinesis and consequently led to bi-/multinucleation. The heavy-chain tails of other kinesin proteins such as kinesin-1 have been shown to have automotor inhibition functions. The binding of proteins or cargos to the tail can release the motor domain for ATP binding and further drive kinesin-1 motility [3, 4]. Therefore, it is possible that MKLP1, as a member of the kinesin family, also operates in a similar way.

### 3.2. Identification of the MKLP1-TD-Interacting Partners by GST Pull-Down and LC-MS/MS Analysis

To further determine the MKLP1 tail domain-binding proteins, we conduct the GST pull-down combined with mass spectrometry analysis. The experiment methods are similar to our previous work [8]. The purified GST and GST-MKLP1-TD proteins are subjected to SDS-PAGE electrophoresis and Coomassie brilliant blue staining; GST and GST-MKLP1-TD show predominant bands as the expected molecular weight (Figure 2(a)). The rat brain lysate supernatants were incubated with prepared GST-MKLP1-TD beads or GST-beads. Followed by adequate washing, the final pull-down proteins are purified and digested with trypsin then analyzed by tandem liquid chromatography-tandem mass spectrometry. The raw data was interpreted with Mascot 2.2 software and retrieve the Uniprot database with a high stringency filtration (score ≥ 20). The identified unique peptides were shown in supplementary table 1 and 2. In which the enriched GST, KIF23 (MKLP1), and trypsin peptides proved that we express the correct GST-MKLP1-TD fusion protein. For the functional overview of the identified partner proteins exist only in the GST-MKLP1-TD pull-down group, we carry out function annotation by GO analysis in Metascape [12] and cellular component or biology process analysis by FunRich software [13]. Biology process analysis results showed that most GST-MKLP1-TD pull-down proteins are involved in the cell division process which corresponds to the function of MKLP1 (Figure 2(b)). Cellular component analysis results showed that those proteins are mainly localized in the nucleus similar to MKLP1's location (Figure 2(c)). In Figure 2(d), GO analysis indicates the most relevant and significant enriched terms (*p* < 0.01). Here, 47 of 54 proteins were annotated in the database and listed in the supplementary table 3. There was a report that key mitotic regulators are controlled through ubiquitylation and proteasome-mediated degradation [14]. Our results also show a significant involvement of ubiquitination modification-related proteins like Ubl7, FBXO40, RNF123, and FBXW10. These proteins should be considered to have an important role on MKLP1 rapid degradation processes and are in line with MKLP1's function in regulating cell division. “String” is a protein interaction database, which contains known and predicted protein interactions (https://string-db.org/). The String database drew a PPI (protein-protein interaction) map based on 54 MKLP1-TD-binding proteins (Supplementary Fig 1) we found. We can intuitively find that among the 54 proteins only three known MKLP1-binding proteins (ZWILCH, RCC2, and CNTRL) are all nuclear proteins. We also found that the ubiquitination-related proteins bind to each other. And most of the remaining proteins have not been reported to bind to MKLP1. Because some reports had proposed that kinases can regulate the kinesin motor activity by phosphorylation [5, 15, 16]. Then, we focused our research on the only one serine-threonine kinase PAK2, which is specifically pulled down by MKLP1-TD.

### 3.3. PAK2 Binds to MKLP1 and Associates with Midbody Components during Cytokinesis

PAK2 is ubiquitously expressed in mammalian tissues and cell lines [17] and had been reported to regulate cell division process [18, 19]. The interaction was further confirmed by immunocytochemistry staining and coimmunoprecipitation experiments. Immunocytochemistry staining of endogenous PAK2 in HEK293 cells from anaphase to cytokinesis (Figure 3(a)) demonstrated that PAK2 was concentrated at the midbody. The spatial and temporal similarities between PAK2 and MKLP1 indicate a possible involvement of PAK2 in the maintenance of the microtubule bundles at the central spindle and organization of the midbody matrix [11, 20]. To further illustrate a relationship between MKLP1 and PAK2 in living mammalian cells, a biophysical approach based on FRET was utilized. MKLP1 and PAK2 were fused with CFP and YFP, respectively, at the C-terminus and were cotransfected into HEK293 cells. To measure the steady-state FRET, the cells cotransfected with different fusion proteins at a ratio of 1 : 1 were imaged using three-channel fluorescence microscopy through the CFP, YFP, and FRET filter channels. The FRET efficiency was quantified as the FR (see Materials and Methods). To ensure that our recording system could reliably detect FRET, controls were set in parallel. As shown in Figures 3(c) and 3(d), cells coexpressing CFP and YFP, which served as negative controls, showed no FRET with FR = 1.01 ± 0.04 (*n* = 15 analyzed cells). However, cells coexpressing the CFP-YFP concatemer, a positive control for FRET, showed the maximum FR (FR = 3.87 ± 0.05 (*n* = 13 analyzed cells)). There was a significant increase in the FR of cells coexpressing PAK2-YFP and MKLP1-CFP (FR = 2.21 ± 0.16 (*n* = 20 analyzed cells)), suggesting that MKLP1 can interact with PAK2 directly in living mammalian cells. By immunoprecipitation assays, we confirmed the interaction between these endogenous proteins. Furthermore, the interaction seemed to be altered according to the cell cycle phase. As shown in Figure 3(b), the association between MKLP1 and PAK2 was intensified during cytokinesis compared with prometaphase, strongly suggesting functional coordination of these proteins during cytokinesis.

### 3.4. Knockdown of PAK2 in 293 Cells Causes Bi-/Multinucleation

To clarify the function of endogenous PAK2 in the progression of cytokinesis, an RNA interference approach was adopted to knockdown PAK2 expression. A PAK2 shRNA-expressing construct and a scrambled control construct were introduced into cultured HEK293 cells (using western blot methods to verify the PAK2 shRNA efficiency and specificity, see Supplementary Fig 2), and the cells were analyzed by immunofluorescence 2 days later. As shown in Figures 4(a) and 4(b), the knockdown of PAK2 by RNA interference resulted in a significantly increased proportion of bi-/multinucleated cells, in contrast to cells transfected with the scrambled shRNA. To make sure this shRNA is specific, we also cotransfected with an increasing amount of PAK2 rescue plasmids (1 : 2), we found that the PAK2 knockdown effect can be rescued, which makes sure this PAK2 shRNA is specific (Figures 4(a) and 4(b)). This cytokinetic defect shared characteristics identical to those resulting from overexpression of the MKLP1 tail domain. Given the association between PAK2 and MKLP1, it is highly possible that the interaction might be of functional significance during cytokinesis.

### 3.5. PAK2 Is Required for Maintaining MKLP1 Localization at the Midbody, and the Knockdown of PAK2 in 293 Cells Causes Cytokinesis Failure

Growing evidence has indicated that some kinesin proteins can be phosphorylated at the tail domain by serine/threonine-protein kinases, leading to changes in the motility of these proteins [15, 16, 21]. Interestingly, PAK2, a serine/threonine kinase, recognizes the consensus sequence (K/RRXS) [22], which exists in the tail domain of MKLP1 (AA804-808, KRRSS). Therefore, PAK2 could be expected to have a regulatory effect on MKLP1's motility, possibly through phosphorylation. To determine whether the association of PAK2 with the tail domain of MKLP1 affects the distribution of MKLP1 during cell division, HEK293 cells transfected with PAK2 siRNA, scrambled RNA, or a pEGFP vector (control) were examined by MKLP1 immunostaining. As shown in Figure 4(c), in control, scrambled, and PAK2 shRNA plus rescue plasmids transfected cells, MKLP1 concentrated predominantly in the midbody during cytokinesis, whereas its localization in cells with siRNA knockdown PAK2 was significantly different. In PAK2 knockdown cells, MKLP1 failed to accumulate at the midbody and dispersed in the daughter cells. These results indicate that the concentration of MKLP1 in the midbody during cytokinesis is PAK2 dependent. It has been reported that the knockdown of endogenous MKLP1 via RNAi affects the formation of the midbody matrix in dividing cells, causing the abnormality of midzone microtubules and resulting in failed cytokinesis [11]. Therefore, proteins that affect the localization and motility of MKLP1 would be expected to impact cytokinesis. Consistent with this idea, we observed that the progression of cytokinesis was impeded by PAK2 knockdown. We transfected cells with scrambled or PAK2 siRNA, by which control cells had fully complete cytokinesis (data not shown). However, microscopy of cells in which PAK2 was knocked down by shRNA showed that, although the cells had attempted cytokinesis, the daughter cell bodies remained connected by a cytoplasmic bridge. After 360min, the cleavage furrow finally regressed and left the daughter cells conjoined as bi-/multinuclear cells (Figure 4(d)).

In summary, we have presented evidence that the tail domain of MKLP1 has an autoinhibitory effect on its own motility and that the interaction of PAK2 with MKLP1 further regulates the motility of MKLP1, consequently affecting the progression of cytokinesis. These observations provide a molecular basis for the regulation of MKLP1 motility during cytokinesis.

## Figures and Tables

**Figure 1:** The tail domain of MKLP1 is crucial for its localization and function during cell division. (a) Schematic diagram showing full-length MKLP1 and its mutants. (b, c) F-MKLP1 concentrates in the nucleus when expressed in HEK293 cells. *Δ*C16-MKLP1 and MSD-MKLP1 showed a higher degree of binding with microtubules and accumulated at the leading edge of the cells compared with the control cells. The arrowheads show accumulated eGFP. Scale bar, 25 *μ*m. (d) HEK293 cells were transfected with plasmid DNA encoding TD-MKLP1 or STD-MKLP1 as indicated. Forty-eight hours after transfection, the cells were fixed, and eGFP and DAPI were detected to allow quantification of the number of mutant-expressing cells, which exhibited a bi-/multinuclear phenotype. (e) The results represent the mean (±S.E.M.) from 3 independent experiments. The overexpression of the MKLP1 tail domain resulted in a significant increase in the numbers of binuclear cells (*p* < 0.01).

**Figure 2:** Bioinformatic analysis for the functional annotation of the predicted MKLP1-TD-associated candidates. (a) Coomassie blue staining to confirm the successful expression and purification of GST-MKLP1-TD and GST (control) proteins. (d) GO analysis shows the most relative and top enriched terms for the identified MKLP1-TD-interacting proteins, individually according to biological process (b) and cellular component (c). The significance of the enriched pathway represented by the number of the -Log10 (*p* value); the ratio of the gene number to each pathway's total number is shown as % in the horizontal axis.

**Figure 3:** PAK2 interact with MKLP1. (a) Synchronised HEK293 cells were fixed and stained for PAK2.The image shows a cell at anaphase and cytokinesis. PAK2 is localized to the spindle midzone (anaphase) and to the midbody (cytokinesis) at the center of the furrow, similar to the localization of MKLP1. (b) Immunoprecipitation (IP) shows endogenous MKLP1 interacting with PAK2 in HEK293 cells. Tubulin was used to normalize the inputs. IB, immunoblot. (c) Transient expression of the CFP and YFP fusion proteins in HEK293 cells, and images are shown by the CFP (A), YFP (B), and FRET (C) channels. FRET^C^ is calculated as described in Materials and Methods and is represented as a pseudocolor. A.l.u.f.i.: arbitrary linear units of fluorescence intensity. Bar, 20 *μ*m. (d) FR values were obtained from individual HEK293 cells expressing the indicated fusion proteins. Data are shown as the mean ± S.E.M and originate from three independent experiments. ^∗∗^*p* < 0.01 versus HEK293 cells cotransfected with CFP and YFP (negative control). Student's *t*-test.

**Figure 4:** Knockdown of PAK2 in HEK293 cells causes cytokinesis failure and bi-/multinucleation. (a) HEK293 cells were transfected with PAK2 shRNA, PAK2 shRNA plus PAK2 rescue plasmid, or scrambled shRNA as indicated. Forty-eight hours after transfection, the cells were fixed, and eGFP and DAPI were detected to allow the quantification of eGFP-expressing cells, which exhibited a bi-/multinuclear phenotype, Scale bars, 30 *μ*m. (b) The results represent the mean (±S.E.M.) from 3 independent experiments. The knockdown of PAK2 resulted in a significant increase in the numbers of bi-/multinucleated cells (*p* < 0.001). (c) HEK 293 cells grown on coverslips were transfected with pEGFP empty plasmid, scrambled shRNA, PAK2 shRNA, or PAK2 shRNA plus PAK2 rescue plasmid. At 48 h after transfection, the cells were fixed and stained with MKLP1 antibodies (red) and DAPI (blue). Scale bars, 10 *μ*m. (d) HEK 293 cells were treated for 2 days with PAK2 shRNA, and microscopy revealed that the living cells attempted cytokinesis but failed. Scale bars, 30 *μ*m.

## Data Availability

The data used to support the findings of this study are available from the corresponding author upon request.

## Supplementary Materials

Supplementary 1 Supplementary Figure 1: the PPI (protein-protein interaction) map based on GST-MKLP1-TD-specific pull-down 54 proteins analyzed by the String database. Supplementary Figure 2: using western blot methods to verify the PAK2 shRNA efficiency and specificity. HEK 293 cells were transfected with scrambled shRNA or PAK2 shRNA. 48h after transfection, the cells were lysated and subject to western blot experiment.

Supplementary 2 Supplementary Table 1: GST pull-down.

Supplementary 3 Supplementary Table 2: GST-MKLP1-TD pull-down.

Supplementary 4 Supplementary Table 3: MKLP1-TD-specific binding protein.
